RETRACTED

# Combination of Methotrexate and Leflunomide Is Efficient and Safe for 60 Patients with Rheumatoid Arthritis

**DOI:** 10.1155/2022/6829358

**Published:** 2022-10-03

**Authors:** Fang Chen, Yingfang Wang, Liuqing Wang, Hongwei Du, Shan He

**Affiliations:** Department of Rheumatology and Immunology, Affiliated Jinhua Hospital, Zhejiang University School of Medicine, Jinhua, Zhejiang 321000, China

## Abstract

The present work is aimed at exploring the clinical efficacy and safety of methotrexate (MTX) and leflunomide (LEF) combination therapy for rheumatoid arthritis. From June 2019 to June 2021, a total of 120 individuals with rheumatoid arthritis received a diagnosis. Sixty patients each were randomly assigned to the control and observation groups. The observation group received MTX and LEF combo medication while the control group only received MTX treatment. Clinical efficacy, complication incidence, and the alleviation of inflammatory markers, joint pain, and clinical symptoms were compared between the 2 groups. Posttreatment, the observation group had overall response rate of 96.66%, while the control group had 86.67%, with significant differences. Compared with pretreatment, both control and observation group patients showed decreasing trends of IL-1 levels and increasing trends of IL-10 levels posttreatment, with significant differences (*P* < 0.05). Compared with the control group, patients in the observation group had lower IL-1 and TNF-*α* levels with significant differences (*P* < 0.05) and higher levels of IL-10 with significant difference (*P* < 0.05). In both groups, the pain score and the number of painful joints were much lower than they were prior to treatment. Following treatment, the observation group displayed significantly lower levels of erythrocyte sedimentation rate, rheumatoid factor, and C-reactive protein than the control group (*P* < 0.05). Clinical measures in the observation group were all lower than those in the control group with statistically significant differences (*P* < 0.05). Moreover, the incidence rate of adverse reactions showed no significant difference between these 2 groups (*P* > 0.05). In conclusion, the combination therapy of MTX and LEF is efficacious for rheumatic arthritis.

## 1. Introduction

Rheumatoid arthritis (RA) is an immune-mediated systemic disease, with chronic, progressive, and symmetrical polyarthritis as cardinal symptom [1]. It is characterized by synovitis and bone erosion induced by joint injury, cartilage destruction, and osteoclast activation, which cause destruction and even deformity of the bone, cartilage, and tendons at last [1]. As the condition worsened, RA can develop ankylosis or other deformities, which could then result in loss of function—one of the key factors in lost productivity and disability among people. In China, there is a 0.2–0.4% prevalence of RA, with a higher incidence in women than in males [2, 3]. The pathogenesis of RA remains unclear and may be related to various factors. Therefore, drug is mainly used for clinical treatment [4]. Although there is no radical treatment, immunosuppressant and biological agents are effective in treatment [5].

RETRACTED

Methotrexate (MTX) was originally designed in the 1940s as a folate antagonist for treatment of various cancers [6]. In the management of early and established RA, MTX is recommended as a first-line drug by the European League Against Rheumatism (EULAR) and the American College of Rheumatology (ACR) [7]. However, it has no significant effect and is accompanied by different side effects [8]. Leflunomide (LEF) is a relatively low-toxic immunomodulator with anticell proliferation and immunosuppressive effects [9]. Recent clinical trials have demonstrated the excellent therapeutic benefit of combining MTX and LEF therapy for RA [10]. To further analyze the efficacy and safety of this combination therapy, we reviewed the clinical materials from 120 cases of RA patients treated in our hospital from June 2019 to June 2021.

## 2. General Clinical Data and Methods

In this paper, we define the general clinical data, methods, and statistical analysis in detail.

### 2.1. General Clinical Data

A total of 120 RA patients who received treatment between June 2019 and June 2021 were chosen as study participants; they all had varying degrees of morning stiffness, pain, and joint swelling, but no connective tissue illnesses, an immunosuppressive drug history, or major somatic diseases. A total of 120 patients were randomly assigned to the control and observation groups (*n* = 60). Control group: 19 males and 41 females, age 43 to 75, mean age 57.6 ± 5.8, 13 elbow cases, 28 shoulder cases, and 19 knee cases; observation group: 16 males and 44 females, age 42-76, mean age 56.9 ± 6.0, 20 elbow cases, 25 shoulder cases, and 15 knee cases. There was no significant difference in general data between the 2 groups (*P* > 0.05), which is comparable when treated with different methods. The Affiliated Jinhua Hospital Ethical Committee of Zhejiang University School of Medicine gave its approval for this study.

### 2.2. Methods

Prior to separate treatment, all patients from the 2 groups received basic treatment, such as health education, joint immobilization, low-dose hormones (methylprednisolone 4 mg once daily), and folic acid (5 mg).

Only once a week for three consecutive months, 7.5 to 10 mg of MTX was administered to the control group. The observation group underwent MTX and LEF combination therapy for three consecutive months, receiving the same dosage of MTX as the control group and 20 mg of LEF once week.

RETRACTED

### 2.3. Outcome Measures

1. Efficacy evaluation: (I) remarkably effective: the patient's clinical symptoms were significantly relieved after treatment. (II) Effective: the patient's clinical symptoms were relieved to some extent after treatment. (III) Ineffective: the patient's clinical symptoms did not change or worsened after treatment. Overall response rate = remarkably effective + effective
2. Improvement of clinical symptoms: the number of swollen joints and sensitive joints, as well as the length of morning stiffness, was examined and recorded before and 4, 8, and 12 weeks following therapy
3. Improvement of the inflammation: the IL-1, IL-10, and TNF-*α* levels in peripheral blood in patients before and after 12 weeks of treatment
4. Visual analogue scale (VAS) was used to assess whether there was joint tenderness. The number of tender joints was counted
5. The occurrence of adverse reactions (nausea, vomiting, oral ulcer, and elevated transaminase) was compared between the 2 groups
6. Comparison of experimental measures: C-reactive protein (CRP), erythrocyte sedimentation rate (ESR), and rheumatoid factor (RF) were compared between the 2 groups

### 2.4. Statistical Analysis

SPSS 20.0 was used for data analysis. Measurement data were expressed as −*x* ± *s*, with line *t*-test as comparison between groups. Enumeration data were expressed as *n* (%), with *χ*^2^ test as comparison between groups. *P* < 0.05 indicated statistically significant difference.

## 3. Results

### 3.1. Clinical Efficacy

Three months after treatment, the clinical efficacy of the 2 groups was evaluated. The total response rate was 96.66% in the observation group and 86.67% in the control group. The data comparison between the 2 groups showed statistically significant differences (*P* < 0.05). The results are shown in Table 1.

### 3.2. Improvement of Inflammation in the 2 Groups

After treatment, the control group showed lower IL-1 level, higher IL-10 level, and lower TNF-*α* level, with statistically significant differences (*P* < 0.05). The observation group also showed lower IL-1 level, higher IL-10 level, and lower TNF-*α* level after treatment, with statistically significant differences (*P* < 0.05). Comparing the two groups, the observation group showed lower levels of IL-1 and TNF-*α* with significant differences (*P* < 0.05) and higher level of IL-10 with significant difference (*P* < 0.05). These results are shown in Figure 1.

### 3.3. Changes of Pain in the 2 Groups

In both groups, the VAS and the number of tender joints after treatment were significantly reduced than before with significant differences (*P* < 0.05), as shown in Figure 2.

RETRACTED

### 3.4. Comparison of Experimental Measures between the 2 Groups

The ESR, CRP, and RF before treatment showed no significant difference between the 2 groups (*P* > 0.05). After treatment, the observation groups showed lower ESR, CRP, and RF than the control group with significant differences (*P* > 0.05). These results are shown in Figure 3.

### 3.5. Changes in Clinical Symptoms in the 2 Groups

Before treatment, there was no significant difference in clinical measures between the 2 groups (*P* > 0.05). Three months after treatment, the clinical measures in the observation group were lower than that in the control group, with significant differences (*P* < 0.05). These results are shown in Figure 4.

### 3.6. Adverse Reactions in the 2 Groups

Control group: cases of nausea and vomiting: 5 (8.33%). Cases of oral ulcer: 2 (3.33%). Cases of elevated transaminase: 2 (3.33%). Observation group: cases of nausea and vomiting: 4 (6.67%). Cases of oral ulcer: 3 (5.00%). Cases of elevated transaminase: 4 (6.67%). The incidence of adverse reactions showed no significant difference between the 2 groups (*P* > 0.05). These results are shown in Table 2.

## 4. Discussion

RA is a chronic syndrome with higher incidence rate in women than in men. The clinical data of both groups in this study were consistent with the characteristics of RA patients, mainly developed from transient and mild pauciarthritis to rapid progressive polyarthritis, involving the wrist, elbow, shoulder, knee, and toe joints, and probably also involving the cervical, temporomandibular, sternoclavicular, and acromioclavicular joints, with limited activity [1]. Arthritis often presents with symmetry, persistent swelling and tenderness, and morning stiffness. Its harm includes causing anemia easily, of which the degree is related to disease activity and joint inflammation degree [11, 12], and causing rheumatoid nodules. Nodules can occur in or around the joint, or subcutaneously, or in any internal organs, commonly inducing pericarditis and secondary Sjogren's syndrome, manifested as dry eyes, dry mouth, saliva, tears, etc. [13]. It is also simple to develop vasculitis, which can affect any part and primarily affects small and medium vessels. The condition has long been the focus of clinical interest because of its devastating effects on patients' lives and careers. Controlling joint and tissue inflammation, symptom relief, maintaining joint function, preventing deformity, and joint healing to relieve pain and restore function are the main goals of treatment [14–16].

RETRACTED

MTX is the most widely used basic drug for RA. It inhibits purine synthesis by inhibiting dihydrofolate reductase, thus inhibiting thymidine synthesis, reducing neutrophil chemotaxis, and inhibiting the release of inflammatory cytokines [17]. Low dose of MTX can significantly ameliorate joint symptoms and the abnormity of various clinical measures [18]. Adverse reactions include anorexia, nausea, vomiting, alopecia, hematocytopenia or thrombocytopenia, drug-induced interstitial pneumonia, damage of liver and kidney function, etc.

LEF is a relatively low-toxic immunomodulator with anticell proliferation and immunosuppressive effects. LEF has been approved by the US Food and Drug Administration as the first oral treatment for RA [19]. Studies have shown that its working mechanism is to inhibit cell adhesion and tyrosine kinase activity, thus affecting the conduction of cell activation [19]. Its active metabolite A771726 selectively blocks the de novo synthesis pathway by inhibiting dihydrolactate dehydrogenase activity in mitochondria, thus interfering with the pyrimidine metabolism, blocking T cells and B cell proliferation, and reducing the production of immunoglobulin [20]. Scholars have also found that LEF inhibits the production of macrophage inflammatory mediators in the synovium. Because the two drugs act on different parts of the immune process, there are synergistic immunosuppressive effects from the mechanism of action [21]. It has been shown that their combination therapy can suppress TNF-*α*, IL-1, IL-6, COX1, COX2, and NK-KB expressions in RA synovial tissues, thus reducing inflammation and improving the patient's condition [22, 23]. It has been suggested that the combination therapy has better efficacy than LEF alone, but with more severe gastrointestinal response and liver toxicity. Some foreign studies believed that the hepatotoxicity of LEF is no more serious than other antirheumatic drugs [24–26]. However, the combination therapy of these two drugs will combine their adverse reactions, too, and as the course of treatment prolongs, the adverse reactions aggravate. Common adverse reactions are nausea, stomatitis, diarrhea, alopecia, rash, and liver injury, with bone marrow suppression appeared on a few patients, occasionally with visible lung interstitial lesions.

In this study, the combination therapy of LEF and MTX was used as treatment for RA patients. The levels of IL-1, IL-10, and TNF-*α* in peripheral blood samples were observed. According to studies, there were substantial disparities between the response rates of the observation group (96.66%) and the control group (86.67%) (*P* < 0.05). Thus, the combination therapy had more obvious efficacy than MTX alone. After treatment, the IL-1 levels were significantly lower than before, with lower levels in the observation group than in the control group, indicating that the combination therapy had a better anti-inflammatory effect on RA patients than MTX alone. IL-10 levels were both greater after treatment in the two groups. The IL-1 and TNF-*α* levels in the observation group and the control were significantly reduced than before, while their levels in the observation group were significantly lower than that in the control group. The reasons may be insufficient dose or treatment course, and the sample size should be increased.

RETRACTED

## 5. Conclusion

In conclusion, the results of this study established that the combination therapy of LEF and MTX had relatively ideal efficiency as treatment for RA. However, this study is a retrospective analysis, which is likely to cause some deviations in the results. It needs to be further confirmed by multicenter clinical trials.

## Figures and Tables

**Figure 1:** Improvement of inflammation in the 2 groups. The levels of IL-1, IL-10, and TNF-*α* in the observation group and the control group were detected. ^∗^*P* < 0.05; #*P* < 0.05, compared with the control group.

**Figure 2:** Changes of pain in the 2 groups. The VAS and the number of tender joints in the observation group and the control group were detected. ^∗^*P* < 0.05; #*P* < 0.05, compared with the control group after treatment.

**Figure 3:** Comparison of experimental measures between the 2 groups. The values of ESR, CRP, and RF in the observation group and the control group were detected. ^∗^*P* < 0.05, compared with the control/observation group before treatment; #*P* < 0.05, compared with the control group after treatment.

**Figure 4:** Changes in clinical symptoms in the 2 groups. The clinical symptoms in the observation group and the control group were detected. ^∗^*P* < 0.05; #*P* < 0.05, compared with the control group after treatment.

**Table 1:** Clinical efficacy of the 2 groups.

Group	*N*	Remarkably effective	Effective	Ineffective	Overall response
Observation	60	32 (53.33)	26 (44.33)	2 (3.34)	58 (96.66)
Control	60	24 (40.00)	28 (46.67)	8 (13.33)	52 (86.67)
*X* ^2^		4.573	1.026	5.157	4.116
*P*		0.001	0.757	0.001	0.002

**Table 2:** Adverse reactions in the 2 groups.

Group	*N*	Oral ulcer	Elevated transaminase	Vomiting	Adverse reactions
Observation	60	3 (5.000)	4 (6.670)	4 (6.670)	11 (18.330)
Control	60	2 (3.330)	2 (3.330)	5 (8.330)	9 (15.00)
*X* ^2^		5.144	2.019	4.472	4.116
*P*		0.431	0.757	0.191	0.257

## Data Availability

The original data used to support the findings of this study are available from the corresponding author upon request.
